RETRACTED

# Different Associated Aspects That Influence Complication Rates on Clinical PKP Surgery Using Smart Medical Big Data

**DOI:** 10.1155/2022/8432360

**Published:** 2022-03-21

**Authors:** Bin Fu, Yi Dong, Fang Xiang, Gen Xia, Zhaohao Ning, Huiqiang Ding

**Affiliations:** ^1^Department of Spinal Orthopedics, General Hospital of Ningxia Medical University, Yinchuan 750000, China; ^2^The Third People's Hospital of Ningxia Hui Autonomous Region, Yinchuan 750000, China

## Abstract

Osteoporotic vertebral compression fractures are on the rise in modern society due to the aging population, and this often results in painful symptoms and kyphotic abnormalities in patients. Bone cement was injected into the vertebral body to reinforce the vertebral body and restore most of the damaged vertebrae's natural height. Percutaneous kyphoplasty is the name given to this type of procedure (PKP). Bone cement leakage has been linked to several problems, according to the research. Neurological problems might arise if bone cement leaks into the spinal canal or the nerve root canal during surgery. As a result, PKP surgeons must now deal with the issue of reducing bone cement leakage. Using smart medical big data, this paper examines a sample of PKP operations and then examines different associated aspects that influence complication rates in order to better advice clinical PKP surgery use. There were 172 vertebral bodies in total in 72 patients receiving PKP surgery at a Chinese hospital that were examined by smart medical big data for vertebral degeneration and fusion. Bone cement leakage and variations in preoperative average anterior vertebral column height, preoperative Cobb angle, and the volume of injected bone cement were considered when dividing the patients into leakage and nonleakage groups; then, we figure out what is causing the bone cement to leak. Five patients experienced lung-related problems out of the 18 vertebral bodies with bone cement leaking that were selected for study. That leakage rate was 10.5%. The differences between the two groups in terms of vertebral compression and bone cement injection were statistically significant based on a single-factor analysis. Bone cement leakage in PKP surgery has been linked to the amount of bone cement injected and whether the vertebral body's peripheral wall was injured, according to multivariate analysis. Lung-related problems are more common in patients with a prior history of illness. Osteoporotic vertebral compression fractures can be successfully treated with percutaneous kyphoplasty. An important risk factor for bone cement extravasation in PKP surgery is the amount of bone cement injected, as well as its viscosity and whether damage to the vertebral body's peripheral wall has occurred.

RETRACTED

## 1. Introduction

Osteoporosis-related vertebral compression fractures are among the most common side effects. Traditional surgical therapy entails vertebral body decompression and different internal fixes to meet the goal of regaining the length of the vertebral body and maintaining the spine's stability. The surgical procedure is very traumatic and seriously affects the patient's quality of life. In this case, percutaneous vertebroplasty (PVP) and percutaneous kyphoplasty (PKP) came into being, and they have been widely used clinically [1–4]. PKP surgery has a wide range of applications. Although the number of accumulated surgical cases is increasing and the technology of surgical operations is becoming more and more mature, the issues created by bone cement leakage are increasingly rising, which has increasingly attracted the attention of clinicians.  Figure 1 is schematic diagram of bone cement filling effect. The mechanism of pain relief of this type of surgery is not fully understood, but mechanically stabilizing the affected vertebral body seems to be the most likely mechanism for pain relief. Studies have shown that percutaneous kyphoplasty can not only quickly alleviate patients' discomfort symptoms but also can effectively reestablish the vertebral body's compression length and correct kyphosis, and its surgical complications are less than traditional percutaneous. Vertebroplasty has obvious advantages and has been widely used in recent years. Due to these advantages of PKP surgery, it has been rapidly developed at home and abroad. Studies have also shown that the postoperative VAS score, Oswestry function score, the height of the injured vertebrae, and the Cobb angle are significantly improved compared with preoperatively. A vast number of studies have found that percutaneous kyphoplasty has a great therapeutic impact in the treatment of osteoporotic spinal compression fractures, but the related complications caused by PKP surgery are also a difficult problem in clinical work, which restricts it to a certain extent.

It is found that the viscosity of the bone cement is low at 5–7 minutes after the preparation of the bone cement. If it is injected at this time, more than 50% of the bone cement leaks immediately after the injection, and the viscosity of the bone cement at 7–10 minutes after the preparation is in the intermediate transient state, less than 10% of the bone cement slowly oozes out after injection, and the bone cement is dough-like and has high viscosity 10 minutes after preparation. Baroud et al. established an experimental model of bone cement leakage in vertebroplasty for compression fractures [5, 6]. By injecting different doses and different viscosities of bone cement into the model, they observed the effects of bone cement leakage and injection dosage and bone cement viscosity [7–9]. No leakage occurs during injection. In addition, he also observed bone cement leakage. The leakage rate is positively related to the injected dose. Since the viscosity of bone cement cannot be assessed objectively, and the cause of bone cement leakage is obvious, our paper did not include the analysis of related factors. In the analysis of several indicators in this research, the dose of bone cement injection and the peripheral wall of the vertebral body are the main risk factors, which affect bone cement leakage in PKP surgery. The preoperative Cobb angle, fracture freshness, vertebral operation site, and surgical approach have no significant effects on bone cement leakage [10]. At present, there is no report on the related factors affecting PKP surgery complications. This article uses smart medical big data to screen the data records of patients who have undergone PKP surgery in a Chinese hospital, analyzes a set of PKP operations, and then analyzes the various factors that affect PKP complications. Related factors could better guide the clinical application of PKP surgery.

RETRACTED

## 2. Related Work

Osteoporosis-related vertebral compression fractures are among the most frequent health problems. Vertebral bodies are more prone to compression fractures than hip and ankle joints, which not only cause acute or chronic pain symptoms but also increase the mortality of patients [11]. Therefore, vertebral compression fractures caused by osteoporosis have received more and more attention. In 1984, French interventional radiologists Galibert and Deramond and others performed percutaneous vertebroplasty (PVP) for the first time. Under X-ray monitoring, polymethylmethacrylate (PMMA) was injected percutaneously into the C2 vertebral body to treat hemangioma. The caused vertebral body destruction relieved the patient's long-term pain. Later, Ducplesnel applied vertebroplasty for the first time to treat vertebral compression fractures caused by osteoporosis and achieved good clinical treatment results. At present, vertebroplasty has been widely used at home and abroad to treat osteoporotic vertebral compression fractures, vertebral angioma, vertebral metastases, myeloma, etc., and have achieved good clinical results. However, current research shows that PMMA has the following shortcomings: (1) PMMA has low biocompatibility and cannot be degraded and replaced by bone. Togawa et al. observed that a fibrous layer was formed at the interface between PMMA and bone, and there were foreign body macrophages and giant cells around the fibrous layer [12]. These cells contained bone cement and barium sulfate particles, which may be related to clinical embolism. There is a certain relationship. (2) The high temperature generated during PMMA polymerization may cause thermal damage to nerve roots and surrounding tissues [13]. (3) Unpolymerized monomers have cardio and pulmonary toxicity. Experiments show that PMMA can increase pulmonary artery blood pressure and reduce lung function, while slowing down heart rate and reducing cardiac output, and increasing the probability of pulmonary embolism. (4) Some patients have inflammatory reaction and transient pain aggravation. In addition, domestic reported a case of spinal cord infarction during vertebroplasty in a patient with vertebral compression fracture caused by multiple bone metastases of lung cancer [14]. Some intraoperative and postoperative complications of PVP have a special relationship with PMMA. Therefore, scholars are currently actively researching some new bone cement materials to replace PMMA, including calcium phosphate cement (CPC), calcium sulfate cement (CSC), strontium-containing bioactive bone cement, and some other new materials. Among them, CPC is currently the most researched and is the most promising biodegradable bone cement material. CPC consists of two parts: solid phase and liquid phase. When used, the two are mixed into a paste, and the fluidity before solidification can be used to fill bone defects of any shape. It has low toxicity, longer curing time, sufficient modulation and injection time, less heat release during curing, and basically no burns to surrounding tissues; has the role of guiding osteogenic crawling substitution; and has good compatibility with surrounding tissues. It can recover the length and biomechanical strength of the damaged vertebral body and can cause obvious inflammation [15]. A three-year follow-up study [16] showed that there is no significant difference between CPC and PMMA in relieving patient pain and maintaining vertebral body stability, but CPC has good biological compatibility and can be gradually replaced by new bone tissue. Therefore, it may replace PMMA in vertebroplasty.

RETRACTED

A variety of documents show that only a small amount of bone cement can restore the stiffness of the compressed vertebra to the level before the injury. But, when continuing to increase the dose significantly improves the stiffness, it will have an impact on the adjacent vertebrae. The same dose of bone cement was injected into the thoracic and lumbar vertebrae. The results showed that the strength of the two groups of vertebral bodies can be restored, but only the stiffness of the thoracic vertebrae can be restored. The role of the injection dose has a certain relationship. Through a retrospective analysis of 158 PVP patients, Kaufmann et al. found that the injection dose of bone cement during PVP surgery was not significantly related to the treatment effect. On the contrary, the more bone cement injected, the more complications it caused. In PKP surgery, if the injected dose of bone cement exceeds the maximum dose that the cavity formed by balloon inflation can hold, the pressure in the vertebral body will suddenly increase [17], which increases the probability of bone cement leakage. Therefore, some scholars believe that in the kyphoplasty, the injection dose of bone cement should be adapted to the degree of balloon expansion during the operation, and the balloon is an indication for the termination of the expansion.

Voggenreiter [18] observed 87 patients treated with balloon vertebroplasty, a total of 145 compressed vertebrae; after the operation, the recovery of the physiological curvature of the spine was observed by CT and the VAS score was used to judge the postoperative pain relief rate. It was found that the balloon dilatation vertebroplasty can restore the normal physiological curvature of the spine and relieve the pain of the patient. Gaitanis et al. [19] performed biomechanical measurements on thoracic vertebrae specimens, and the results showed that balloon expansion under physiological preload can significantly correct vertebral deformities and shift the axial load force line back to reach the anterior arrangement of the vertebral body. Reduce the additional flexion moment of the vertebral body moving forward on the adjacent vertebral body by the axial load force line of the vertebral body, thereby reducing the risk of refracture of the adjacent vertebral body. Eck [20] synthesized 168 different types of literature on the efficacy of PVP and PKP surgery and found that both can relieve patients' pain symptoms, but PKP can effectively reduce the leakage rate of bone cement and reduce new compression fractures. Villarraga's study [21] showed that the pressure and tension of the adjacent vertebral body are minimal during percutaneous kyphoplasty, and it was found that the pressure and tension at the level of the vertebral body for treatment are higher than the limit that cortical bone and cancellous bone can tolerate. It is believed that subsequent fractures have nothing to do with surgery. Although percutaneous kyphoplasty has many advantages, the expansion balloon used in the operation is expensive, and PVP and PKP are effective for fresh vertebral compression fractures, but for old vertebral compression fractures. Fractures, due to the lack of space required for forming, can often cause bone cement leakage, which can easily cause serious complications. In response to the shortcomings of PKP and PVP, Israel Disc-O-Tech has developed an expandable vertebroplasty, which can be easily inserted into the vertebral body percutaneously without excessively destroying the vertebral body structure. After it is in the proper position in the vertebral body, the vertebral body is compressed and expanded. When the height of the compressed vertebral body is restored, the Sky shaper is taken out, and bone cement is injected into the formed vertebral body cavity to strengthen the vertebral body to maintain the height of the vertebral body. Zheng et al. [22] treated 25 patients with a total of 30 vertebral compression fractures by using the Sky Shaper. They found that they had good pain symptoms, improved spinal motor function, and restored the height of the compressed vertebral body. The only shortcoming was that it still could not avoid the leakage of bone cement. In order to overcome the problem of bone cement leakage caused by the above three surgical methods, Taiwan A-Spine company developed a new type of Vessel-X bone material filler percutaneous vertebroplasty system on the basis of the kyphoplasty system. The dense polymer mesh structure that constitutes the Vessel-X bone material filler can wrap most of the bone cement and allow an appropriate amount of bone cement to leak out of the mesh layer to anchor with the surrounding bone tissue and Vessel-X during surgery. The bone material filler does not need to be withdrawn. Therefore, this type of operation can not only better control the distribution of bone cement in the vertebral body but also avoid the possibility of bone cement leakage, thereby improving the safety of the operation. Both cadaver specimen studies [23] and preliminary clinical applications [24] have shown the above advantages, but the feasibility and safety of the exact clinical application require further clinical studies. In summary, percutaneous vertebroplasty is a safe and effective method for treating vertebral compression fractures [25]. However, there are still some shortcomings, and further research is needed to improve it for better performance.

RETRACTED

## 3. Methods

### 3.1. General Information

72 cases of osteoporotic vertebral compression fracture patients who underwent PKP surgery were screened by smart medical big data, aged 51–90 years old, with an average age of 70.5 years, of which 18 were males and 54 were females, with a total of 172 vertebrae from T4 to L5, and each patient involves 1 to 7 vertebrae. According to the recorded clinical manifestations, the symptoms of lower back pain of varying degrees, which aggravate after activities, cannot be relieved even in severe cases; the corresponding spinous process tenderness and percussion pain are positive, with or without history of trauma; and the duration of symptoms is 1 to 11 months with an average of 5.8 months. All cases had no symptoms and signs of spinal cord and nerve root damage, and the results of conservative treatment were not satisfactory [26]. Laboratory examinations and systemic examinations confirmed that there were no obvious surgical contraindications.

### 3.2. Imaging Examination

According to the big data recorded prior to the surgery, the spine X-ray film, MRI, and CT examination of the vertebral body were taken routinely. MRI examination uses high-resolution 1.5 T MR imager (SIEMENS MAGNETOM Symphony). The spin echo sequence is used in the sagittal T1 weighted picture, whereas the fast spin echo sequence and fat suppression sequence are used in the T2 weighted picture [27]. All X-ray examinations showed that the vertebral body was osteoporotic with some vertebral body height loss, and some vertebral body compression fractures showed wedge-shaped deformation [28]. MRI examination ruled out other vertebral body diseases and was diagnosed as an osteoporotic vertebral body compression fracture. CT scan of the vertebral body determines whether the peripheral wall of the patient's vertebral body is intact. Three days after operation and during follow-up, X-rays of the spine were routinely examined to understand the reduction of the fractured vertebral body, the distribution of bone cement, and the leakage.

### 3.3. Bone Density Measurement

The bone mineral density (BMD) assessed using MEDILINK's OSTEOCORE-3 DEXA, a French-made device. Osteoporosis can be diagnosed based on WHO diagnostic criteria. Bone density is lower than the average value of normal young adults, −2.5 standard deviations; that is, *T* ≤ −2.5 SD is diagnosed as osteoporosis.

### 3.4. Surgical Methods

All operations are performed by the same team. The patient is in the prone position, the chest and the anterior superior iliac spine are raised to make the abdomen suspended, general or local anesthesia is selected according to the patients' overall condition, and the United States is adopted through the unilateral or bilateral pedicle approach under the fluoroscopy positioning of the C-arm X-ray machine Kyphon's minimally invasive devices and special balloons to perform percutaneous kyphoplasty [29]. During the operation, the balloon expansion and fracture reduction were observed by the C-arm X-ray machine. When the vertebral body reduction was satisfactory or the balloon expansion pressure increased significantly, the balloon was stopped and taken out, and the bone cement prepared into toothpaste state was injected into the vertebral body. Postoperative patients routinely take third-generation bisphosphonates, active Vitamin D, calcium carbonate, and anti-osteoporosis Chinese medicine.

RETRACTED

### 3.5. Evaluation Index

1. Measure the pain intensity VAS and Oswestry function before operation, 3 days after operation, and during follow-up after operation. Score (0–45 points), observe the patient's pain relief and functional recovery. Here, VAS is visual analog scale, 0–10 points, 0 points as painless, and 10 points as the most painful.
2. Pre- and postoperative side medical imaging of the spine shows to measure the anterior edge and midheight of the vertebral body and the Cobb point on the lateral radiographs using a scale, and calculate the average value of the anterior border and midheight of the vertebral body before and after surgery [30]. The average height of the anterior and middle column of each vertebral body is measured. The Cobb angle is measured using the Phillips method, which is based on standard lateral X-rays taken before and after the operation with the diseased vertebrae as the center, measuring from the top end plate of a vertebral body to the diseased vertebra. The Cobb angle of the inferior end plate of the next vertebral body is defined as the “local sagittal cobb angle” (local sagittal cobb angle) [31]. For multiple vertebral compression fractures, if the diseased vertebrae are connected, measure a common local sagittal Cobb angle; if the diseased vertebrae are not connected, measure their local sagittal Cobb angles separately. The change of the local sagittal Cobb angle can reflect the height restoration of each bad vertebral body and the degree of correction of kyphotic deformity. Two spine surgeons who were not engaged in the procedure took all the measures, and the average between the two doctors' measurement results was taken as the final result for analysis and research.
3. According to the MRI signal changes in the fractured vertebrae, it is divided into two types, and two imaging physicians classify each diseased vertebra according to the two types, respectively. If there are differences in classification, discuss with the third imaging physician. A consensus was reached, and the classification criteria are as follows: fresh type: T1WI and T2WI signals are evenly distributed in the vertebral body. A low signal on T1WI, a strong signal on T2WI, and a STIR pattern that progressively transitions from normal bone marrow are all signs of this condition. Subfresh type: the signals on T1WI and T2WI are unevenly distributed in the vertebral body and are distributed in patches, spots, or strips. The signal changes are not uniform, manifested as T1WI, low signal mixing, T2WI and STIR sequences, and low and high signals mixing.
4. Divide the patients into leakage group and nonleakage group whether there is bone cement leakage, and analyze the preoperative average height of the anterior vertebral column, preoperative Cobb angle, bone cement injection volume, and fracture freshness between the two groups. Whether there is a difference in degree, unilateral and bilateral pedicle approach, vertebral body operation site, and whether there is bad for the peripheral wall of the vertebral body, relevant factors that affect the bone cement leakage of PKP surgery can be judged. The statistical processing was processed by relevant statistical software, and the data were expressed as (*x* ± *s*). The single-factor analysis was conducted by *t*-test and *X*^2^ test, and the logistic regression technique was used for the multivariate analysis.

RETRACTED

## 4. Experiments and Discussion

### 4.1. Diagnosis Results

A total of 172 vertebral bodies in 72 patients underwent PKP surgery, all of which fully tolerated the surgery. No nerve or spinal cord injury or balloon rupture occurred during the operation. Intraoperative bleeding was 25–55 ml, with an average of 40 ml. Lie supine for 7 hours after surgery, sit up after 13 hours, and move on the ground 24 hours later. According to the records, the follow-up time was 8 to 18 months, with an average of 14 months. The VAS score, Oswestry function score, and vertebral body height were obviously improved on the 3rd day after surgery and during the follow-up after surgery.  Table 1 shows surgery results of all selected objects.  Figure 2 shows comparison of various indexes before and after operation/continuous nursing.  Figure 3 displays the *t* value comparison of various indexes.

Leakage group: bone cement leakage occurred in 18 vertebral bodies, with a leakage rate of 10.5%, of which 8 cases leaked to the paravertebral body, 7 cases leaked out of the intervertebral space, 2 cases leaked along the pedicle needle route, and 1 case of spinal canal with a small amount of leakage inside. The remaining 154 vertebrae were included in the nonleakage group. Each observation index is summarized in Table 2.  Figure 4 shows comparison of indicators between the leakage group and the nonleakage group.  Figure 5 presents the *t* value comparison of various indexes.

### 4.2. Experimental Results and Analysis

Univariate analysis showed that the differences in the degree of vertebral compression, the number of bone cement squirt, and the presence or absence of vertebral wall damage between the disclosure and the nonleakage groups were statistics obviously, while they are no significant distinct in the preoperative Cobb angle, fracture freshness, vertebral body operation site, and surgical approach of all the patients. The consequence of multivariate research indicated that the amount of bone cement injected and whether extravertebral wall is destroyed are the main factors leading to bone cement leakage in PKP surgery. In all patients, 5 patients had postoperative pulmonary complications, and one of them was diagnosed as cemented pulmonary embolism.  Figure 6 presents chest radiograph showing multiple tubular opacities.  Figure 7 presents multislice spiral CT pulmonary angiography.  Figure 8 presents chest CT showing some high-density intracavitary cement.  Figure 9 presents summary of characteristic and quality of lung-related complications.

RETRACTED

### 4.3. Discussion

All patients with pulmonary complications have a history of pulmonary disease, so such patients are more prone to pulmonary complications. A total of 10 vertebral body compression fractures occurred in 7 patients, 7 of which were adjacent vertebral bodies, but there was no obvious discomfort and was not treated. The rest of the patients did not have new compression fractures, the morphology of the vertebral body did not change significantly, and the height was maintained satisfactorily.

The injection dosage of bone cement in clinical operation is a long-term controversial issue. A variety of documents show that only a small amount of bone cement will recover the stiffness of the compressed vertebra to pre-injury degree. But, when continuing to increase the dose significantly improves the stiffness, it will have an impact on the adjacent vertebrae. Belkoff made 144 vertebral compression fracture models on 12 cadavers, and the results showed that the injection of 2 ml of bone cement can restore the spinal column's toughness, while regaining the stiffness of the vertebral body needs 6 ml in the lumbar spine and 8 ml in the thoracolumbar segment. There were 8 times of bone cement revelation in the experiment, and all cases occurred in cases where 6 ml or more was injected. Clinical studies have confirmed that the amount of bone cement squirt is not connected to the analgesic effect clinically. On the contrary, the more the bone cement injected, the more the complications caused.

In this paper, the average bone cement injection dose of the leakage group was 5.34 ml, which exceeded the 4.17 ml of the nonleakage group. This result also confirmed the above conclusion. In PKP surgery, increased pressure in the vertebral body due to bone cement squirt may lead to cement revelation if the injected dosage is more than what can be held in the cavity created by balloon inflation. Therefore, the injection should not be overemphasized to fill the entire vertebral body with bone cement, and the dose should be adapted to the size of the cavity created by the expanding of the balloon. The indications for the termination of balloon expansion include the following: the height of the vertebral body returns to normal; although there is no height recovery, the balloon has expanded to the endplate; the balloon touches one lateral cortex; the pressure of the balloon no longer decreases during expansion; and the maximum pressure or volume of the balloon has been reached. The volume is used as an estimate of the amount of bone cement injected. It can reach the clinical effect and also decrease the extravasation of bone cement. If a vertebral body fracture has been caused by osteoporosis and the surrounding tissue has been damaged, the risk of surgery increases due to the easy revelation of bone cement; in particular, the back wall damage of the vertebral body has been listed as a contraindication for surgery. The surgical technique uses PKP surgery to treat osteoporotic vertebral body fractures with damaged peripheral vertebral body walls. If the anterior wall of the vertebral body is damaged, then use bone cement to infuse in stages, and if the posterior or side wall of the vertebral body is damaged, then use the full-course dynamic “C” arm. The X-ray machine monitors the perfusion process, effectively preventing the leakage of bone cement and avoiding complications. It should be noted that bone cement leakage is more likely to occur during PKP surgery for osteoporotic vertebral fractures with damaged peripheral walls, which is 33.3% in this group of cases. At the same time, the surgeon must have rich experience and proficient surgical skills. An analytical paper found that the probability of PKP surgery causing pulmonary embolism is 0.3%. Although the probability of occurrence is small, once it occurs, the consequences are quite serious. The vertebral body is composed of loose bone, bone pith, and fat tissue. The bone pith and fat tissue are located in the bone tissue space directly connected to the venous system in the vertebral body. Since there is no valve tissue in the vertebral venous system, and the syringe of bone cement into the vertebral body requires a greater injection pressure, the tissue and bone cement may enter the abundant venous plexus in the vertebral body under such high pressure. When the cement is still in a low-viscosity state, its fluidity is large, and it is easier for the blood to flow back into the extravertebral venous plexus and into the upper and lower vena cava system connected to it. If emboli enter the lungs with blood circulation, it may cause bone cement pulmonary embolism and cause clinical symptoms. In severe cases, respiratory failure may occur, leading to death. The clinical symptoms may be caused by bone cement, and chemical damage induces increased pulmonary capillary permeability and small blood vessel inflammation, thereby releasing inflammatory mediators. Inflammatory mediators cause continuous increase in pulmonary arteriole pressure. In our paper, it was found that 4 patients with postoperative pulmonary complications all had different degrees of pulmonary disease before surgery. Due to the reduced lung function of these patients, pulmonary symptoms and even triggering are more likely to occur under the stimulation of inflammatory mediators, pulmonary embolism. Another related paper found that the occurrence of pulmonary complications after PKP is related to the treatment of multiple vertebral bodies at the same time. However, because there are fewer cases of pulmonary complications in our paper, it is not enough to draw in conclusion. As the accumulated number of cases increases, we will also conduct further research on this issue.

RETRACTED

## 5. Conclusion

In summary, the reasons for bone cement leakage can be summarized as follows: (1) the bone cement has low viscosity, relatively large fluidity, and easy penetration, leakage into the adjacent tissue structure; (2) there are fracture cracks in the severely compressed vertebral body; and (3) continuous injection of excessive bone cement causes relatively higher pressure in the vertebral body. Therefore, clinically, CT or MRI must be performed before PKP surgery to determine whether the spinal body's outer wall has been damaged. Personal surgical methods are utilized for osteoporotic spinal fractures with compromised outer wall. The entire operation process should be closely monitored under X-ray fluoroscopy. It should not be overemphasized that the entire vertebral body should be full of bone cement during injection; in addition, timing of bone cement syringe needs to be grasped. If the syringe is too early, the bone cement has low viscosity and relatively fluidity. Larger and prone to leakage, it should be injected when the bone cement becomes doughy, so as to minimize the occurrence of leakage complications. In addition, strict control of the operation stage and routine application of anti-osteoporosis medications after PKP are necessary measures to prevent postoperative fractures. Since this paper is not based on a small number of samples screened by smart medical big data, and the probability of complications in PKP surgery is low, there are fewer cases in the leakage group, which may reduce the validity of the comparative analysis, and further need to be done. A large sample studies have verified the conclusion. It is hoped that this study will arouse attention to the relevant factors affecting the complications of PKP surgery, so as to reduce the complications caused by PKP surgery.

RETRACTED

## Figures and Tables

**Figure 1:** Schematic diagram of bone cement filling effect.

**Figure 2:** Comparison of various indexes before and after operation/continuous nursing.

**Figure 3:** The *t* value comparison of various indexes.

**Figure 4:** Comparison of indicators between the leakage group and the nonleakage group.

**Figure 5:** The *t* value comparison of various indexes.

**Figure 6:** Chest radiograph showing multiple tubular opacities.

**Figure 7:** Multislice spiral CT pulmonary angiography.

**Figure 8:** Chest CT showing some high-density intracavitary cement.

**Figure 9:** Summary of characteristic and quality of lung-related complications.

**Table 1:** Surgery results of all selected objects.

Item	Before surgery	After surgery	Consecutive	*t*	*p*
VAS	7.8 ± 1.1	2.6 ± 0.8	2.8 ± 1.1	10.4	<0.01
Oswestry function	41 ± 2.8	20 ± 2.5	21 ± 1.1	16.7	<0.01
Cobb angle (◦)	22.8 ± 4.3	12.9 ± 7.7	13.0 ± 7.8	4.2	<0.02
Vertebral height (mm)	16.4 ± 4.7	21.3 ± 5.0	20.8 ± 5.2	4.1	<0.03

**Table 2:** Two types of clinical characteristics.

Characteristics	Leakage group	Nonleakage group	Statistic	*p*
Vertebral height (mm)	11.8 ± 4.1	16.4 ± 4.2	*t* = 2.0	0.05
Cobb angle	24.0 ± 6.5	22.8 ± 4.5	*t* = 0.6	0.59
Cement volume	5.3 ± 1.8	4.2 ± 1.7	*t* = 2.5	0.02
Acute fracture	9	79	*X* ^2^ = 0.08	0.78
Subacute fracture	8	76		
Vertebral incompetence	12	23	*X* ^2^ = 21.9	<0.001
Vertebral competence	6	131		
Thoracic vertebra	12	82	*X* ^2^ = 0.24	0.63
Lumbar vertebrae	7	71		

## Data Availability

The simulation experiment data used to support the findings of this study are available from the corresponding author upon request.
